This article has been retracted.

# Analysis of the Role and Mechanism of ZEB1 in Regulating Cervical Carcinoma Progression via Modulating PD-1/PD-L1 Checkpoint

**DOI:** 10.1155/2022/1565094

**Published:** 2022-04-30

**Authors:** Yuhong Lin, Xiaoxian Wang

**Affiliations:** Fuzhou First Affiliated Hospital of Fujian Medical University, Fuzhou City, 350004 Fujian Province, China

## Abstract

**Background:**

Cervical carcinoma (CC) is a common and highly malignant tumor in women. The involvement of zinc finger E-box binding homeobox 1 (ZEB1) in many kinds of tumors has been well-documented; however, its role and mechanism in CC remain to be clarified.

**Objective:**

This study investigated the mechanism of ZEB1 in modulating the growth and metastasis of CC cells.

**Methods:**

The expression of ZEB1 in CC tissues and adjacent normal counterparts was determined by reverse transcription-polymerase chain reaction (RT-PCR). The correlation between ZEB1 and patient clinicopathological indexes was analyzed. In vitro, gain and loss functions of ZEB1 were performed in C-33A and HeLa cell lines. The proliferation, migration, and invasion of CC cells were detected by Cell Counting Kit-8 (CCK-8) assay and transwell assay, respectively. The expression levels of apoptosis-related proteins such as BCL2-associated X (Bax), B-cell lymphoma-2 (Bcl2), and Caspase-3, as well as epithelial-mesenchymal transition (EMT)-associated proteins including E-cadherin, Vimentin, and Snail, were measured by Western blotting. In addition, the targeting relationship between ZEB1 and programmed death 1 (PD-1)/programmed cell death-ligand 1 (PD-L1) was predicted by bioinformatics and further verified by dual-luciferase reporter assay.

**Results:**

ZEB1 was significantly up-regulated in CC tissues compared with normal counterparts. ZEB1 overexpression promoted the migration, proliferation, and invasion of CC cells and inhibited apoptosis, while knocking down ZEB1 contributed to the opposite effects. In addition, experiments on related mechanisms confirmed that ZEB1 targeted the 3'EUTR terminal of PD-1/PD-L1 and negatively regulated its expression. And an interaction between ZEB1 and PD-1/PD-L1 was identified.

**Conclusion:**

ZEB1 can promote the proliferation and metastasis of CC cells via modulating the PD-1/PD-L1 checkpoint.

## 1. Introduction

There are many kinds of female reproductive system cancers, among which cervical carcinoma (CC) is one of the most common malignant tumors with high morbidity and mortality [1]. Human papilloma virus (HPV) is the most important predisposing factor for CC [2]. Surgery, radiotherapy, and chemotherapy are currently the mainstays of treatment for CC. However, because of the absence of specific clinical presentations at the initial stage of CC, the disease has always reached the advanced stage when patients are treated. In addition, the indications for surgical treatment are limited by tumor staging, coupled with serious side effects caused by radiotherapy and chemotherapy, causing serious psychological and physiological impacts on women [3]. Therefore, it is urgent to establish a more effective strategy for early diagnosis and targeted therapy of CC.

Zinc finger E-box binding homeobox 1 (ZEB1) is a major element of the transcription factor network that regulates epithelial-mesenchymal transition (EMT). It has been found that ZEB1 is abnormally expressed in multiple cancers and is considered as an oncogene that promotes cancer migration, invasion, and metastasis [4]. For example, ZEB1 is shown to interact with the growth factor hepatoma-derived growth factor (HDGF) and induces its transcription to promote the invasion and metastasis of endometrial carcinoma [5]. In addition, the tumor protein P73 antisense RNA 1 (TP73-AS1) elevates ZEB1 expression through adsorption of microRNA (miR)-200a, thus promoting the growth of breast cancer [6]. However, the specific regulation mechanism of ZEB1 in CC needs to be further clarified.

Programmed cell death receptor-1 (PD-1) is an immunosuppressant molecule of the CD28 family [7]. PD-1 has two ligands, namely, programmed cell death-ligand 1 (PD-L1) and PD-L2, which are transmembrane molecules belonging to the B7 family. PD-L1 is a transmembrane protein composed of 290 amino acid subunits, and its extracellular segment consists of two immunoglobulin constant (IgC) regions and IgV-like domains. PD-1, as an inhibitory co-receptor, can inhibit the activity of T cells after interacting with PD-L1, making the cells arrest in the G0/G1 phase, thus inhibiting the proliferation and inducing the apoptosis of T cells. In tumor patients, high expression of PD-L1 can enhance the ability of tumor metastasis, leading to increased mortality of patients [8, 9].

In recent years, PD-1/PD-L1 pathway-targeting immunotherapy has shown obvious antitumor effects in a variety of solid tumor patients [10]. Currently, it has been found that ZEB1 promotes the progression and immune escape of diffuse large B-cell lymphoma by regulating the PD-1/PD-L1 immune checkpoint [11]. However, it waits to be clarified whether this feedback loop can affect the EMT of CC by modulating PD-1/PD-L1.

This study aims to explore the effect of ZEB1 on the occurrence and development of CC, especially epithelial to mesenchymal transition-like transformation. Through experimental research, ZEB1 was found to promote the EMT of CC by regulating the PD-1/PD-L1 checkpoint, which provides an important reference for the clinical treatment of CC.

## 2. Materials and Methods

### 2.1. Tissue Specimens

Forty-two CC patients (mean age: 50 years; age range: 31-67) who received surgical treatment in Fuzhou First Affiliated Hospital of Fujian Medical University from October 2017 to October 2018, were enrolled. All patients' case data were complete, and none of them received radiotherapy, chemotherapy, or other antitumor therapy before diagnosis. The cancer tissue and adjacent healthy tissue of the subjects were collected during the operation and frozen for use. All study participants provided written consent. This research was approved by the Research Ethics Committee of our hospital and was conducted in strict accordance with the Declaration of Helsinki.

### 2.2. Cell Culture

Human cervical epithelial (HUCEC) and CC (HeLa, Caski, C-33A, AV3) cell lines, all purchased from the American Type Culture Collection (ATCC; Rockville, MD, USA), were cultured a medium containing 1% penicillin/streptomycin (Invitrogen, CA, USA) +10% fetal bovine serum (FBS; Thermo Fisher Scientific, MA, USA) + Roswell Park Memorial Institute (RPMI) 1640 (Thermo Fisher Scientific, MA, USA) in a 5% CO_2_ and 37°C incubator. Cells during the logarithmic growth phase were digested and passed by 0.25% trypsin (Thermo Fisher HyClone, UT, USA). C-33A and HeLa with significant differences in expression levels were selected as auxiliary research objects.

### 2.3. Cell Transfection

CC cells during the logarithmic growth phase were planted in 6-well plates (5 × 10^6^/well) after digestion and passage and then transfected after the cells grew stably. ZEB1 overexpression plasmids and corresponding control (Vector), as well as ZEB1 knockdown plasmids (Si-ZEB1) and corresponding control (Si-Vector), were transfected into C-33A and HeLa, according to the instructions of FuGENE® HD transfection reagent (Roche, Shanghai, China), and set as ZEB1 group and Si-ZEB1 group, respectively. Cells were cultured in a 5%CO_2_ and 37°C incubator, and the culture medium was changed 6 h after transfection for 48 h of incubation. After total RNA isolation, the transfection efficiency was determined using reverse transcription-polymerase chain reaction (RT-PCR). Successfully transfected cells were used for research.

### 2.4. RT-PTR

Deoxyribonuclease I was used to remove genomic DNA from the TRIzol-isolated total RNA and then came the reverse transcription reaction with the use of a reverse transcription kit (Shanghai Hifun Biotechnology Co., Ltd., China, RT3) following the operation procedures. Reaction conditions: 70°C/10 min; cooling on ice for 5 min; 42°C/60 min; 95°C/5 min and; 0°C/5 min. The fluorescent quantitative PCR reaction system was 25 *μ*L, comprising cDNA template (500 ng), upstream and downstream primers (each 250 nmol/L), and 2×SYBR Green PCRMaster Mix (12.5 *μ*L). Glyceraldehyde-3-phosphate dehydrogenase (GAPDH) was the internal reference. Primer sequences can be found in Table 1. Reaction was then performed by putting the reaction tube into the MX3000P real-time PCR reactor, with conditions described below: 94°C, 55°C, and 72°C, for 45 cycles. Fluorescence signal monitoring was then carried out. 22^(-*ΔΔ*Ct)^ value was used to indicate the gene's relative expression, where Ct represented the number of amplification cycles when the fluorescence signal of the amplified product reached the set threshold during PCR amplification, and ΔΔ represented the sample to be tested (Ct [target gene] - Ct [GAPDH]) - control group (Ct [target gene] -Ct [GAPDH]).

### 2.5. Cell Counting Kit-8 (CCK-8) Assay

Cells of each group (C-33A and HeLa) in exponential growth phase were collected to prepare a single cell suspension. After cell counting and cell density adjusting, cells were planted into 96-well plates with 1000 cells/well. Each group had 6 multiple wells, and the cells were inoculated onto 6-well plates for 12, 24, 48, 72, and 96 hours. After cell adherence, 90 *μ*L medium and 10 *μ*L CCK-8 solution (Beijing Yita Biotechnology Co., Ltd., China, YT8193) were added to the samples. At the same time, a blank control well containing only culture medium and CCK-8 solution was established and incubated for 2 h. The absorbance (A) of each well was measured at 450 nm using a microplate reader (Thermo Fisher Scientific, M A, USA).

### 2.6. Western Blotting (WB)

Total protein of different groups of cells was extracted with the protein extraction kit (Beijing Applygen Technologies Inc., China, P1250-50/100), and the bicinchoninic acid (BCA) method was adopted for concentration determination of proteins. Total protein (50 *μ*g) was loaded on each well after isolation using the sodium dodecyl sulfate polyacrylamide gel electropheresis. Two hours after electrophoresis, the protein was transferred to a polyvinylidene fluoride (PVDF) membrane using the wetting transfer method, followed by 1 h of blocking with 5% skimmed milk, and the subsequent overnight cultivation with primary antibodies BCL2-associated X (Bax) (ab32503), B-cell lymphoma-2 (Bcl2) (ab59348), cleaved Caspase-3 (ab2302), E Cadherin (ab40772), Vimentin (ab92547), SNAIL (ab53519), and ZEB1 (ab185228) all diluted at the ratio of 1 : 1000 and purchased from Abcam, USA. The next morning, the TBS+Tween (TBST; Beijing Yita Biotechnology Co., Ltd., China, YT8022) rinsed membrane was placed into the horseradish peroxidase-labeled secondary antibody goat antirabbit (ab6721, 1 : 3000, USA) for 1 h of incubation at 37°C. This was followed by development with enhanced chemiluminescence (ECL), image acquisition and optical density measurement using the Quantity One (EasyBio (Beijing) Technology Co., Ltd., China). The experiment was repeatedly determined three times.

### 2.7. Cell Migration and Invasion by Transwell Assays

Cells (5 × 10^4^ cells/well) were planted in 24-well culture plates on day 1 and transfected following the Lipofectamine TM2000 instructions on day 2 when the cell density reached about 80%. After 24 h of transfection, cells were seeded into the apical chamber (2.5 × 10^4^ cells/well) and suspended in a serum-free medium. While the medium of basolateral chamber comprised 20% serum, for the migration experiment, there was no Matrigel (Beijing Solarbio Science & Technology Co., Ltd., China, M8370) on the interior of the apical chamber. For cell invasion, a layer of Matrigel-simulated extracellular matrix (final concentration of Matrigel: 2 mg/mL. After attenuation with serum-free culture medium, 40 *μ*L was dripped into each chamber for 30 min to 1 h of standing at 37°C to gel) was prelayered on the inside of the chamber. After 24 h of cell migration and invasion, the chamber was removed. Cells were then fixed with a mixture containing formaldehyde and acetic acid for 15 min, washed with PBS, and dyed with crystal violet. After staining, the cells were rinsed with 1 × phosphate buffer saline (PBS). Cells in the apical chamber were erased with Q-tips, and cell invasion and migration were microscopically observed.

### 2.8. Biological Analysis and Dual-Luciferase Reporter Assay

Through the JASPAR (http://jaspar.genereg.net/) tool, the potential binding site of ZEB1 on the PD-L1 promoter was searched. Si-NC and Si-ZEB1 were co-transfected into C-33A cells. Forty-eight hours after transfection, the luciferase activity was measured with the dual-luciferase assay system.

### 2.9. Chromatin Immunoprecipitation (ChIP) Experiments

C-33A cells were stained with 1% formaldehyde and lysed for 10 min at room temperature. After sonication for 30 min, the genome was fragmented to about 500 bp. Cell lysates were incubated with antibodies for 12 h, and the purified immunoprecipitated chromatin was determined by RT-PCR.

### 2.10. Statistical Analysis

The software used for data analysis was SPSS17.0 (SPSS Inc., Chicago, IL, USA). The quantitative data was expressed as mean ± standard deviation (*X* ± *S*), and the statistical methods for identifying the difference between and among groups were *t*-test and one-way analysis of variance (ANOVA), respectively, with the significance level set at *P* < 0.05.

## 3. Results

### 3.1. Expression of ZEB1 in CC and Its Relationship with TNM

The expression of ZEB1 was not significantly different among patients in different age groups (*P* > 0.05, Table 2). *X*^2^ or rank sum test results showed that the expression of ZEB1 was higher in patients with poorly differentiated tumors than in those with well-differentiated tumors; stage III-IV patients exhibited higher ZEB1 expression than those in stage I-II; ZEB1 expression was higher in cases with lymph node metastasis than in those without; ZEB1 was higher in patients with distant metastasis than in those without. All the above differences were of statistical significance (*P* < 0.05, Table 2). Analysis of clinical specimens showed that the higher the expression of ZEB1, the worse the CC differentiation, the more significant the metastasis, and the higher the TNM stage (Table 2).

### 3.2. Regulation of ZEB1 on CC Cell Proliferation and Apoptosis

RT-PCR was used to measure the expression of ZEB1 in CC tissue and cell lines. ZEB1 expression was found to be significantly elevated in cancer tissues compared with normal counterparts (*P* < 0.05, Figure 1(a)), and ZEB1 was obviously up-regulated in CC cell strains (HeLa, Caski, C-33A, and AV3) compared with HUCEC (*P* < 0.05, Figure 1(b)), suggesting the involvement of ZEB1 in the onset and development of CC. To explore its mechanism, ZEB1 was overexpressed in C-33A and underexpressed in HeLa. CCK8 assay results identified that the proliferation ability of cells overexpressing ZEB1 was up-regulated versus the control group and decreased when ZEB1 was knocked down (*P* < 0.05, Figures 1(c) and 1(d)). WB was used to detect the expression of apoptosis-related proteins. It was found that Bax and Caspase-3 protein levels were down-regulated and Bcl2 protein expression was up-regulated when ZEB1 was overexpressed. After knockdown of ZEB1, the protein expression of Bax and Caspase-3 was up-regulated, and Bcl2 protein expression was down-regulated (*P* < 0.05, Figures 1(e) and 1(f)). Therefore, ZEB1 is up-regulated in CC cells and tissues and can promote tumor cell proliferation and inhibit apoptosis.

### 3.3. ZEB1 Promotes EMT of CC Cells

We used transwell assays to investigate the effect of ZEB1 on the metastasis and EMT of CC cells. Cell migration and invasion levels were significantly up-regulated after ZEB1 overexpression, and the reverse was true after knocking down ZEB1 (*P* < 0.05, Figures 2(a) and 2(b)). In addition, WB results identified decreased E-cadherin and elevated Vimentin and Snail after overexpression of ZEB1 compared with the control group, and the reverse was true when ZEB1 was knocked down (*P* < 0.05, Figure 2(c)). It indicates that ZEB1 enhances the EMT of CC cells.

### 3.4. ZEB1 Transcription Up-Regulates PD-1/PD-L1 Expression and Promotes EMT

We further studied the specific regulation of ZEB1 on PD-1/PD-L1 in CC. Through JASPAR (http://jaspar.genereg.net/), we found that ZEB1 had two binding sites on the PD-L1 promoter (*P* < 0.05, Figure 3(a)). As indicated by RT-PCR and WB, the mRNA and protein levels of ZEB1 and PD-L1 were significantly down-regulated after knocking down ZEB1 (*P* < 0.05, Figures 3(b)–3(d)). According to ChIP assay, DNA fragments containing PD-L1 promoters at locus 1 or 2 were enriched in ZEB1 antibody precipitation (*P* < 0.05, Figure 3(e)). Dual-luciferase assay showed that the luciferase activity of PD-L1 promoter was significantly weakened following ZEB1 knockdown, but the effect was partially reversed by mutations at the locus 1 or 2; however, silencing ZEB1 did not change the luciferase activity of PD-L1 promoter when both loci 1 and 2 were mutated (*P* < 0.05, Figure 3(f)). These results indicate that ZEB1 transcription up-regulates the expression of PD-1/PD-L1.

## 4. Discussion

CC is one of the most serious female reproductive system tumors, which is characterized by high incidence and mortality. Women of all ages are susceptible to CC, especially the middle-aged, seriously affecting their psychological health and social activities [12]. With the rapid economic and social development and the change of people's living habits, the exposure factors of CC are increasing day by day [13]. Surgical resection is the preferred treatment for CC, but a review of the data shows that there is still a certain risk of recurrence after surgery [14]. At present, there are two major bottlenecks in treatment: one is the immature early diagnosis method, and the other is the low survival rate of advanced cancer treatment. Therefore, it is necessary to identify the molecular mechanisms of occurrence and progression of CC as well as the therapeutic targets [15]. Starting from molecular and protein expression and function, this study found through various experiments that ZEB1 could promote the growth and metastasis of CC cells via modulating PD-1/PD-L1, which is of great clinical implications for the early diagnosis of CC and identifying new therapeutic drugs.

PD-1 is a member of the immunoglobulin superfamily, and in CC, PD-1/PD-L1 co-expression predicts unfavorable prognosis [16, 17]. Previous research suggests that ZEB1 acts as a transcription factor to induce EMT in cancer cells to promote tumor progression [18]. The oncogenicity of ZEB1 has been demonstrated in multiple solid tumors such as osteosarcoma, retinoblastoma, and neuroblastoma, which plays a positive regulatory role in the malignant progression of these tumors [19]. ZEB1 also plays a carcinogenic role in CC and regulates the malignant development of CC by mediating the colorectal neoplasia differentially expressed (CRNDE)/miR-4262/ZEB1 signaling pathway [20]. Recent evidence has revealed that ZEB1 regulates the expression of PD-1/PD-L1 in tumor cells and thus affects tumor progression, suggesting that ZEB1 is closely related to PD-1/PD-L1 in tumor development [21]. In addition, highly expressed mucin 1 (MUC1) can activate the nuclear factor-k-gene binding (NF-*κ*B)/ZEB1/PD-L1 signaling pathway, leading to poor prognosis of nonsmall cell lung cancer (NSCLC), while blocking therapy targeting PD-1/PD-L1 can significantly improve NSCLC treatment, suggesting that PD-1/PD-L1 co-expression plays a carcinogenic role in NSCLC [22]. Moreover, Kim S et al. found a significant connection between high expression of ZEB1 and PD-L1 and EMT phenotype in pulmonary adenocarcinoma (PADC), and PD-1/PD-L1 blocking immunotherapy has become a promising therapeutic option for PADC [23].

Interestingly, this study found that ZEB1 was up-regulated in CC, confirming the interaction between ZEB1 and PD-1/PD-L1. It was also found that ZEB1 could bind to the promoter of PD-L1 and activate its transcription to induce the EMT of CC. The results of this study are similar to those of Zhao L et al. [11], but their research focuses on elucidating the effect of the small nucleolar RNA host gene 14 (SNHG14)/miR-5590-3p/ZEB1 feedback loop on the progression and tumor immune escape of diffuse B-cell lymphoma. The novelty of this study is that it is proposed for the first time that ZEB1 and the PD-1/PD-L1 feedback loop only promote tumor cell growth in CC but also significantly affect its EMT.

## 5. Conclusion

To sum up, this research confirms that ZEB1 promotes the progression and EMT of CC in vitro, and clarifies that ZEB1 can accelerate the EMT of CC cells by activating the PD1/PD-L1 immune checkpoint, all of which further suggest the role of ZEB1 as a candidate target gene for immunotherapy of CC, providing a new direction for the development of novel therapies for CC.

## Figures and Tables

**Figure 1:** ZEB1 regulates the proliferation and apoptosis of cervical carcinoma cells. (a)–(b) RT-PCR was used to detect the expression of ZEB1 in cervical carcinoma tissues (*n* = 42) and cell lines. In order to explore its mechanism, ZEB1 was overexpressed in C-33A cells and knocked down in HeLa cells. (c)–(d) CCK-8 assay was used to detect the proliferation of cervical carcinoma cells. (e)–(f) Western blotting was used to detect the expression of apoptosis-related proteins Bax, Caspase-3, and Bcl2. ∗∗ indicates *P* < 0.01, and ∗∗∗indicates *P* < 0.001 compared with HUCEC, Vector, Si-Vector, or between two groups.

**Figure 2:** ZEB1 promotes the EMT of cervical carcinoma cells. (a)–(b) Transwell assay was used to explore the effect of ZEB1 on the metastasis of cervical carcinoma cells. (c) Western bolt experiment was conducted to detect the expression of E-cadherin, Vimentin, and Snail. ∗∗ indicates *P* < 0.01, and ∗∗∗indicates *P* < 0.001 compared with Vector, Si-Vector, or between two groups.

**Figure 3:** ZEB1 transcription up-regulates the expression of PD-1/PD-L1 and promotes EMT. (a) We further studied the specific regulation of ZEB1 on PD-1/PD-L1 in cervical carcinoma and found through JASPAR (http://jaspar.genereg.net/) that ZEB1 has two binding sites on the PD-L1 promoter. (b–d) The mRNA and protein expression of ZEB1 and PD-L1 after ZEB1 knockdown was detected by RT-PCR and Western blotting experiments. (e) ChIP assay was used to analyze the DNA fragment of PD-L1 promoter in the precipitation of ZEB1 antibody. (f) The dual-luciferase assay was used to detect the effect of ZEB1 knockdown on the luciferase activity of PD-L1 promoter. nsP > 0.05; ∗ indicates *P* < 0.05, ∗∗ indicates P <0.01, and ∗∗∗ indicates *P* < 0.001 compared between two groups.

**Table 1:** Prime sequences.

Gene	Forward	Reverse
ZEB1	5′-CCCATTGTCCCCATTTTGCA-3′	5′-AGGCAGCAGGAATCAGTCTT-3′
PD-1	5′-CAGGTTGCTGCGTCCGAGGT-3′	5′-AGTGGACAATAGGTCGGGC-3′
PD-L1	5′-TGCTTCTCAAGTGTGGTCCTAG-3′	5′-CGCGTGAAGGCAGCTATA-3′
GAPHD	5′-TGGTTGAGCACAGGGTACTT-3′	5′-CCAAGGAGTAAGACCCCTGG-3′

**Table 2:** Relationship between the expression of ZEB1 and clinical features in tissue specimens of patients with cervical carcinoma.

Characteristics	Patients	Expression of ZEB1		P-value
		High-ZEB1	Low-ZEB1	
Total	42	16	26	
Age (years)				0.746
<65	15	5	10	
≥65	27	11	16	
Differentiation				0.001∗
Middle or low	21	2	19	
High	21	14	7	
TNM stage				0.002∗
I-II	30	7	23	
III-IV	12	9	3	
Lymphatic metastasis				0.001∗
Yes	15	12	3	
No	27	4	23	
Distant metastasis				0.001∗
Yes	10	9	1	
No	32	7	25	

Note: ∗ indicates *P* < 0.05, namely, the difference was statistically significant.

## Data Availability

The simulation experiment data used to support the findings of this study are available from the corresponding author upon request.
